# Integrative bioinformatics approaches to map key biological markers and therapeutic drugs in Extramammary Paget’s disease of the scrotum

This article has been retracted.

**DOI:** 10.1371/journal.pone.0254678

**Published:** 2021-07-22

**Authors:** Fatima Noor, Muhammad Hamzah Saleem, Jen-Tsung Chen, Muhammad Rizwan Javed, Wafa Abdullah Al-Megrin, Sidra Aslam

**Affiliations:** 1 Department of Bioinformatics and Biotechnology, Government College University, Faisalabad, Pakistan; 2 College of Plant Science and Technology, Huazhong Agricultural University, Wuhan, China; 3 Department of Life Sciences, National University of Kaohsiung, Kaohsiung, Taiwan; 4 Biology Department, Faculty of Science, Princess Nourah Bint Abdulrahman University, Riyadh, Saudi Arabia; Universite d’Orleans, FRANCE

## Abstract

Extramammary Paget’s disease (EMPD) is an intra-epidermal adenocarcinoma. Till now, the mechanisms underlying the pathogenesis of scrotal EMPD is poorly known. This present study aims to explore the knowledge of molecular mechanism of scrotal EMPD by identifying the hub genes and candidate drugs using integrated bioinformatics approaches. Firstly, the microarray datasets (GSE117285) were downloaded from the GEO database and then analyzed using GEO2R in order to obtain differentially expressed genes (DEGs). Moreover, hub genes were identified on the basis of their degree of connectivity using Cytohubba plugin of cytoscape tool. Finally, GEPIA and DGIdb were used for the survival analysis and selection of therapeutic candidates, respectively. A total of 786 DEGs were identified, of which 10 genes were considered as hub genes on the basis of the highest degree of connectivity. After the survival analysis of ten hub genes, a total of 5 genes were found to be altered in EMPD patients. Furthermore, 14 drugs of CHEK1, CCNA2, and CDK1 were found to have therapeutic potential against EMPD. This study updates the information and yields a new perspective in the context of understanding the pathogenesis of EMPD. In future, hub genes and candidate drugs might be capable of improving the personalized detection and therapies for EMPD.

## 1. Introduction

Extramammary Paget disease (EMPD) arises as rare cutaneous adenocarcinoma, accounting small proportion (about 6.5%) of all Paget’s disease cases. The very first time, EMPD was uncovered by Radcliffe Crocker about half a century ago [1–4]. The frequency of occurrence is higher at various anatomical locations such as the scrotum, vulva, and perianal region [5, 6]. In women, the vulvar EMPD accounts for 81.3% of all EMPD cases while scrotal EMPD accounts for 43.2% of all EMPD cases in men [7]. The risk of getting EMPD is increasing 3.2% per year. However, it is unknown why EMPD cases of the scrotum and other anatomic sites are increasing [8, 9]. The overall frequency of hospitalization is common under the age of 65 years [10]. It has a great diversity of clinical symptoms that vary considerably in the context of disease status and prognosis [10, 11]. However, owing to insufficient diagnostic methods, EMPD patients are diagnosed, on average, at the middle or late disease stage, which consequently, leads to a poor prognosis [12, 13]. Hence, the understanding of molecular mechanisms that contributes to the pathogenesis and prognosis of EMPD has become increasingly important for the development of multiple therapeutics and diagnostics approaches.

Until now, EMPD is incurable and dramatically increases the morbidity as well as the mortality rate in developed countries. As the information pileup, the same scenario is predicted in the developing countries [14]. Multiple remedies such as imiquimod, 5% cream, or cytotoxic agent with 1% 5-fluorouracil cream [15, 16] are available but all these revolve around the management of disease, however, the actual treatment is yet to be discovered.

The discovery of potential biomarkers that can halt the pathophysiology of the disease and can act as a virtual shortcut, will be considered as the miracle of the current era. The mind-boggling potential benefits of molecular biomarkers offer multiple innovative perspectives to improve diagnostic as well as treatment options. Several studies were conducted to identify the potential biomarkers for monitoring and diagnosis of EMPD, but all these studies might conflict due to the complicated molecular mechanism of EMPD [17, 18].

Nowadays, the use of bioinformatics is getting popular across all facets of life sciences. Recently, it has been seen as an outbreak of emerging sequencing technologies that enable researchers to make ground-breaking discoveries in the domain of computational biology. In recent decades, bioinformatics along with microarray technologies has paved the way for researchers to identify disease-related genes involved in the pathogenesis of EMPD. Various bioinformatics-related researches on plenty of human diseases had proven reliable and persuasive, so it implies that integrated bioinformatics analysis can contribute to evaluating the underlying complex molecular mechanism of EMPD of the scrotum.

In spite of the numerous studies on EMPD, no sufficient evidence is present yet to prove the existence of disease-related genes, and their involvement in the pathogenesis of EMPD. To tackle this issue, we used integrated bioinformatics approaches to figure out the disease-related functional genes as problem-solving negotiators to switch off the progression of EMPD. Moreover, investigation of drug-genes interactions in the present work can contribute to the discovery of therapeutic candidates for drug repurposing.

## 2. Materials and methods

### 2.1. Retrieval of microarray

Gene Expression Omnibus (GEO) database in National Center for Biotechnology Information (NCBI) is a freely available public database, enclosing the gene profiles [19]. Expression profile of GSE117285 based on GPL17077 platform (Agilent-039494 SurePrint G3 Human GE v2 8x60K array) was retrieved from NCBI-GEO database [20]. Dataset include 4 controls and 4 EMPD cases.

### 2.2. Identification of DEGs

GEO2R is considered as a useful interactive web tool for comparison and analysis of sample of multiple groups [21]. In present study, GEO2R tool was employed to explore the Differential Expressed Genes (DEGs) among controls and EMPD patients of GSE117285 dataset. Genes that satisfy the criteria of |log_2_ (fold change) | > 1.0 and adjusted P-value < 0.05 were distinguished as DEGs. Volcano plot was constructed using ggplot2 package of R, to visualize the significant and non-significant DEGs.

### 2.3. Analysis of DEGs at functional level

At the functional level, a database for annotation, visualization, and integrated discovery (DAVID) was used to perform GO enrichment analysis and KEGG pathway analysis [22]. The DEGs were subjected to DAVID for the prediction of DEGs function at three levels: Biological process (BP), Molecular function (MF), and Cellular component (CC). The top 10 significant items of GO and KEGG pathways were demonstrated in form of bubble maps which were plotted using ggplot2 package of R. In this regard, P<0.05 was believed to be statistically-significant.

### 2.4. Construction of protein-protein interaction network

Search Tool for the Retrieval of Interacting Genes/Proteins(STRING) was used for the functional interactions among DEGs at the combined score of more than 0.5 [23]. Molecular Complex Detection (MCODE) plugin from Cytoscape was utilized for distinguishing the module that best represents the clusters of DEGs [24]. The modules which met the cutoff criteria of node > 10 and the score >10 were selected. Further, the resulted modules were subjected to DAVID for pathway analysis.

### 2.5. Selection of hub genes

CytoHubba plugin was used for distinguishing hub genes among up and down expressed DEGs. A total of twelve topological analysis methods are available in the cytoHubba. Among these 12 methods, the degree method was chosen for the identification of hub genes.

### 2.6. Survival analysis of hub genes

EMPD is a malignant skin cancer characterized by the appearance of Paget cells. GEPIA server was employed to evaluate the expression level of hub genes among Skin Cutaneous Melanoma (SKCM) and normal tissues [25]. In this regard, P-value< 0.05 was believed to be statistically significant.

### 2.7. Drug-gene interaction analysis

Drug-Gene Interaction Database was used to search hub genes against known and potentially small drug-like molecules [26]. The final list was included only FDA-approved drugs. Finally, the STITCH tool was used for the visualization of interaction network among gene and their associated drug candidates [27].

## 3. Results

### 3.1. Identification of DEGs

In the present study, microarray dataset GSE117285 was obtained from Agilent-039494 SurePrint G3 Human GE v2 8x60K Microarray, which consists of 8 samples (4 healthy controls and 4 EMPD patients). A total of 786 DEGs was identified, of which 619 were upregulated genes and 167 were downregulated genes (**S1 Table)**. Moreover, gene differential expressions were presented in form of a volcano map (**Fig 1**).

**Fig 1:** Representation of differential expressed genes in form of Volcano plot with red dots showing upregulated genes while blue dots showing downregulated genes. Black dots represent non-significant genes.

## 3.2. Functional enrichment analysis of DEGs

GO enrichment and KEGG pathways analysis of DEGs were performed to analyze the gene function in terms of biological processes, cellular components, and molecular function as well as their associated pathways. GO enrichment analysis of the top 10 significantly enriched terms showed that in the BP category, the genes involved are concerned with cell division, mitotic nuclear division, cell proliferation, sister chromatid cohesion, organ regeneration, and inflammatory responses (**Fig 2(A)**). In terms of CC, the genes were enriched nucleus, cytosol, nucleoplasm, extracellular space, and centrosome (**Fig 2(B)**). For MF, a category the genes were mainly concentrated in the protein binding, ATP binding, protein kinase activity, protein serine/threonine kinase activity, and chromatin binding (**Fig 2(C)**). KEGG enrichment pathway analysis revealed that genes were significantly enriched in the cell cycle, viral carcinogenesis, Hepatitis B, TNF signaling pathway, and oocyte meiosis (**Fig 2(D)**).

**Fig 2:** Representation of GO enrichment and KEGG pathway analysis. (A) Gene ontology in terms of BP (B) Gene ontology in terms of CC (C) Gene ontology in terms of MF(D) KEGG pathway analysis.

### 3.3. Construction of PPI network and the analysis of DEGs

PPI network of DEGs obtained from STRING were subjected to the MCODE plugin of Cytoscape which provided significant 22 modules. From these modules, the top two functional clusters of modules were selected based on the cutoff criteria of node > 10 and the score is ≥10 (**Table 1**). KEGG pathway analysis of the selected modules revealed that the genes belong to these clusters are enriched in the TNF signaling pathway, toll-like receptor signaling pathway, chemokine signaling pathway, cytokine and cytokine receptor interaction, and complement and coagulation cascades (**Fig 3**).

**Fig 3:** Two modules were selected having cutoff criteria node > 10 and the score is ≥. 10 (A) The first module constructed from MCDOE comprised of 55 genes; (B) Pathways associated with the first module; (C) The second module constructed from MCDOE comprised of 14 genes; (D) Pathways associated with the second modules.

**Table 1:** Top 2 modules were selected having cutoff criteria node > 10 and the score is ≥ 10.

Clusters	Score	Nodes	Edges	Nodes IDs
1	49.296	55	1331	MELK, CCNA2, PLK4, SMC4, KIF23, NCAPG, DLGAP5, MND1, FBXO5, TYMS, RAD51AP1, AURKA, TRIP13, ARHGAP11A, ATAD2, CENPK, CENPN, CENPA, HJURP, ASPM, CEP55, CENPF, PBK, FANCI, KIF2C, CDK1, KIF4A, ECT2, EXO1, KNTC1, HMMR, ERCC6L, HELLS, CDC45, SKA3, FAM83D, BUB1, CHEK1, BIRC5, MAD2L1, CDKN3, BUB1B, STIL, CDCA2, SKA1, SPC25, SPAG5, CENPU, CKS2, CDCA5, CENPE, KIF18A, NDC80, KIAA0101, RAD54L
2	10.615	14	69	MRPL13, RPS4X, MAGOHB, RPL22L1, RPS2, MRPL1, RPS11, PSMA1, RPL7A, EIF2S2, EIF4E, RPL13A, RPS6, RSL24D1

### 3.4. Selection of hub genes

Using 12 methods available in the cytoHubba, the topmost ten genes were selected and ranked by degree method. These ten genes named CDK1, MAD2L1, BUB1, CCNA2, BUB1B, NCAPG, NDC80, KIF2C, CENPF, and CHEK1 were considered as the hub genes (**Fig 4**). Moreover, the interaction network of hub genes to their related neighboring genes is shown in **Fig 5.**

**Fig 4:** (A) Construction of PPI network of 6 hub genes (B) Observed coexpression of 10 hub genes in Homo sapiens.

**Fig 5:** Interaction network of genes to their related neighboring genes.

### 3.5. Survival analysis of hub genes

GEPIA server was used for the survival analysis of 10 hub genes. The survival analysis of 10 hub genes revealed 5 significant genes (**Fig 6**). These 5 genes named CHEK1, KIF2C, CENPF, CCNA2, and CDK1 were demonstrated as significant because of the p-value <0.05. Moreover, the expression level of 5 genes varied significantly among SKCM and normal tissues.

**Fig 6:** Survival analysis of CHEK1, KIF2C, CENPF, CCNA2, and CDK1 in GEPIA server.

### 3.6. Drug-gene interaction

A total of 14 drugs were explored using DGIdb that might have the potential to treat PD patients. CHEK1, CCNA2, and CDK1 were chosen as possible targets of 14 drugs based on the DrugBank source (**Table 2**). Furthermore, using the STITCH tool, downstream interaction networks of CHEK1, CCNA2, and CDK1 were generated (**Fig 7**).

**Fig 7:** (A) Targetable CHEK1 subnetwork. (B) Targetable CCNA2 subnetwork. (C) Targetable CDK1 subnetwork.

**Table 2:** List of FDA approved drugs.

Search_ term	Match_ term	Match_ type	Gene	Drug	Interaction_types	Sources	Pmids
CHEK1	CHEK1	Definite	CHEK1	PALBOCICLIB		DTC	
CHEK1	CHEK1	Definite	CHEK1	CISPLATIN		CIViC	28490518
CHEK1	CHEK1	Definite	CHEK1	OLAPARIB		CIViC	28490518
CHEK1	CHEK1	Definite	CHEK1	GEMCITABINE		NCI	17245119
CHEK1	CHEK1	Definite	CHEK1	FOSTAMATINIB	inhibitor	DrugBank	26516587
CHEK1	CHEK1	Definite	CHEK1	ETOPOSIDE		DTC	22364746
CCNA2	CCNA2	Definite	CCNA2	TAMOXIFEN		PharmGKB	24622579
CDK1	CDK1	Definite	CDK1	SERTRALINE		DTC	16680159
CDK1	CDK1	Definite	CDK1	RUCAPARIB		DTC	
CDK1	CDK1	Definite	CDK1	FENOFIBRATE		DTC	16680159
CDK1	CDK1	Definite	CDK1	CINNARIZINE		DTC	16680159
CDK1	CDK1	Definite	CDK1	CLOFIBRATE		DTC	16680159
CDK1	CDK1	Definite	CDK1	FOSTAMATINIB	inhibitor	DrugBank	26516587
CDK1	CDK1	Definite	CDK1	CLOTRIMAZOLE		DTC	16680159

## 4. Discussion

EMPD is considered a rare malignant dermatosis with poorly defined outcomes [28, 29]. Clinically, the more frequent indication of EMPD is eczematous [30]. There has been substantial heterogeneity regarding various EMPD cases that lead to the earlier detection, a thought-provoking question [31–33]. Recently, a comprehensive study on patients suffering from EMPD has made it clear that progress in the overall pathogenesis of EMPD varies from patient to patient which turned the diagnosis as well as treatment of EMPD into a challenging task [34]. The current work planned to identify the disease-related functional genes involved in the progression of EMPD in the scrotum. This whole research revolves around the analysis of gene ontology, gene enrichment pathways, PPI, and hub genes. The gene expression microarray profiles of the GSE117285 dataset were analyzed using integrated bioinformatics analysis. Through KEGG pathway analysis, the DEGs were significantly found to be enriched in the cell cycle, viral carcinogenesis, Hepatitis B, TNF signaling pathway, oocyte meiosis, RIG I like receptor signaling pathway, Legionellosis, and NOD-like receptor signaling pathway. Our functional annotation of target genes might be helpful in understanding this targeted slicing on the pathogenesis of EMPD. In the current work, after the survival analysis of ten hub genes, a total of 5 genes were found to be altered in EMPD patients involving CHEK1, KIF2C, CENPF, CCNA2, and CDK1. Hence, it represents that these genes plays important role in the pathogenesis of EMPD. Furthermore, 14 drugs of CHEK1, CCNA2, and CDK1 were found to have therapeutic potential against EMPD.

CHK1 kinase is considered a key element of DNA damage response. There is no study available regarding the role of CHK1 in EMPD. Apoptosis is caused when DNA damage is extremist. Recently a study has shown that Chk1 inhibition encourages cancerous cells to undergo apoptosis and inappropriately arrest damaged DNA [35]. CHK1 plays important role in tumor suppression hence might prove fruitful to combat the disease condition by preventing EMPD from becoming malignant. By targeting CHK1, the pathogenic mechanisms of EMPD can be controlled, hence might serve as a molecular biomarker for the diagnosis and treatment of EMPD.

Cyclin-dependent kinase 1(CDK1) is a key member of the CDKs family, crucial for the cell cycle progression [36, 37]. During the last ten years, a slew of studies has made it clear that CDK1 encourages tumor growth as well as enables cancerous cells to proliferate spontaneously [38, 39]. According to previous reports, CDK1 has been implicated in the development of various cancers, such as liver and colorectal cancer [40–42]. EMPD is considered a rare cancer-related disease and found to have an association with skin cancer [43]. Hence all this evidence provides a precious clue that upregulation of CDK1 might control the intricate molecular mechanism behind the progression of EMPD.

CCNA2 is considered a therapeutic target in skin cancer [44]. Multiple studies on CCNA2 has made it clear that upregulation of CCNA2 interfere the normal process and leads to proliferation of cancerous cell spontaneously [45]. During the process of the cell cycle, CCNA2 regulates G1/S as well as G2/M transitions. It was discovered to be a prognostic biomarker for melanoma survival [44, 46]. Hence by considering CCNA2 as a molecular biomarker, the diagnosis and treatment of EMPD might become an easy task. Considering our analysis, we propose that the upregulation of CCNA2 might induce EMPD.

Identification of aberrant pathways in EMPD patients might reveal the molecular mechanism underlying and uncover more enthralling and promising molecular candidates with effective diagnostic and prognostic value. KEGG pathway analysis of CHEK1, CCNA2, and CDK1 revealed that this gene disturbs the cellular pathways through disruption in cell cycle and p53 signaling pathway which unfortunately leads to the disease condition. It is noteworthy that CHEK1, CCNA2, and CDK1 are involved in cell cycle regulation. Cancer is an unregulated cell division caused by the failure in cell cycle regulation. EMPD is malignant skin cancer, hence these findings conclude that EMPD interferes with the regulatory mechanism of the cell cycle and contributes to the development of skin cancer. These findings shed light on the pathogenesis of EMPD and facilitate the development of personalized treatment for EMPD. The disturbed pathways identified using integrated bioinformatics analysis may have an important role to play in the pathogenesis of EMPD. Additional studies are required to investigate the molecular mechanisms behind these aberrant pathways and EMPD development.

## 5. Conclusion

In the present work, a mechanism was proposed to explain the progression in the pathogenesis of EMPD. It might due to the genes that disturb the cellular pathways which ultimately leads to the disease condition. This research discerned hub genes as key biological markers and their associated pathways involved in the development of EMPD. Based on our knowledge, CHEK1, CCNA2, and CDK1 have not been previously reported to be related to EMPD. It was found that these genes might act as potential biomarkers for the diagnosis of EMPD at an early stage. Our findings reveal that EMPD causes disruption in cellular pathways which unfortunately makes the disease condition much worse. In the near future, further study and clinical trials are required for the identification of genes and small drug-like molecules having effective diagnostic and prognostic value, respectively. Our research will serve as a significant pioneer for the researchers who want to identify the associated pathways involved in the pathogenesis of EMPD. This research relies on various freely available databases to shed light on EMPD pathogenesis and treatment. *In vivo* and *in vitro* investigations of genes and pathways interaction are essential to delineate the specific roles of the identified genes, which could confirm gene functions and reveal the mechanisms underlying EMPD. In the future, additional experimental research on these hub genes could lead to an increase in our knowledge to fight against EMPD by means of novel therapeutic approaches. Based on the hub genes, experimental models may be designed in terms of the detection of pathogenesis, evaluation of risk, and determining the targeted therapies of EMPD.

## Supporting information

S1 Table List of upregulated and downregulated DEGs. (DOCX)

## References

[1] WagnerG, SachseMM. Extramammary Paget disease–clinical appearance, pathogenesis, management. JDDG: Journal der Deutschen Dermatologischen Gesellschaft. 2011;9(6):448–54. doi: 10.1111/j.1610-0387.2010.07581.x 21205169

[2] TulchinskyH, ZmoraO, BrazowskiE, GoldmanG, RabauM. Extramammary Paget’s disease of the perianal region. Colorectal Disease. 2004;6(3):206–9. doi: 10.1111/j.1463-1318.2004.00630.x 15109389

[3] LiY-C, LuL-Y, YangY-T, ChangC-C, ChenL-M. Extramammary Paget’s disease of the scrotum associated with hepatocellular carcinoma. J Chin Med Assoc. 2009;72(10):542–6. doi: 10.1016/S1726-4901(09)70425-3 19837650

[4] St ClaireK, HooverA, AshackK, KhachemouneA. Extramammary paget disease. Dermatol Online J. 2019;25(4). 31046904

[5] SimondsRM, SegalRJ, SharmaA. Extramammary Paget’s disease: a review of the literature. Int J Dermatol. 2019;58(8):871–9. doi: 10.1111/ijd.14328 30569580

[6] DelportES. Extramammary Paget’s disease of the vulva: an annotated review of the current literature. Australas J Dermatol. 2013;54(1):9–21. doi: 10.1111/j.1440-0960.2012.00898.x 22671146

[7] ZhouS, ZhongW, MaiR, ZhangG. Mammary and extramammary Paget’s disease presented different expression pattern of steroid hormone receptors. BioMed research international. 2017;2017. doi: 10.1155/2017/3768247 29082243PMC5610822

[8] WrightJL, MorganTM, LinDW. Primary scrotal cancer: disease characteristics and increasing incidence. Urology. 2008;72(5):1139–43. doi: 10.1016/j.urology.2008.06.043 18799208

[9] HerrelLA, WeissAD, GoodmanM, JohnsonTV, OsunkoyaAO, DelmanKA, et al. Extramammary Paget’s disease in males: survival outcomes in 495 patients. Ann Surg Oncol. 2015;22(5):1625–30. doi: 10.1245/s10434-014-4139-y 25384700

[10] LamC, FunaroD. Extramammary Paget’s disease: summary of current knowledge. Dermatol Clin. 2010;28(4):807–26. doi: 10.1016/j.det.2010.08.002 20883922

[11] LeeSJ, ChoeYS, JungHD, AhnSK, ChaYC, ChoKH, et al. A multicenter study on extramammary Paget’s disease in Korea. Int J Dermatol. 2011;50(5):508–15. doi: 10.1111/j.1365-4632.2010.04661.x 21506963

[12] LingH, HuX, XuX-L, LiuZ-B, ShaoZ-M. Patients with nipple-areola Paget’s disease and underlying invasive breast carcinoma have very poor survival: a matched cohort study. PLoS ONE. 2013;8(4):e61455. doi: 10.1371/journal.pone.0061455 23620755PMC3631229

[13] ChandawarkarRY, RicchuitiD, AmjadI, MarsicoREJr, WellsMD. Extramammary Paget’s disease of the perineum: Avoiding pitfalls in diagnosis and management. Canadian Journal of Plastic Surgery. 2003;11(4):205–8. doi: 10.1177/229255030301100406 24009439PMC3760750

[14] YinS, XuL, WangS, FengJ, LiuL, LiuG, et al. Prevalence of extramammary Paget’s disease in urban China: a population-based study. Orphanet J Rare Dis. 2021;16(1):1–7. doi: 10.1186/s13023-020-01625-z 33731175PMC7972239

[15] BermanB, SpencerJ, VillaA, PoochareonV, ElgartG. Successful treatment of extramammary Paget’s disease of the scrotum with imiquimod 5% cream. Clin Exp Dermatol. 2003;28:36–8. doi: 10.1046/j.1365-2230.28.s1.12.x 14616812

[16] LiuR, WeiX, WeiH, HuB. Case Report Extramammary Paget’s disease of the scrotum: a case report and review of the literature. Int J Clin Exp Med. 2017;10(12):16750–4.

[17] GatalicaZ, VranicS, KrušlinB, PoormanK, StaffordP, KacerovskaD, et al. Comparison of the biomarkers for targeted therapies in primary extra‐mammary and mammary Paget’s disease. Cancer medicine. 2020;9(4):1441–50. doi: 10.1002/cam4.2820 31899853PMC7013075

[18] BarthP, Dulaimi Al-SaleemE, EdwardsKW, MillisSZ, WongY-N, GeynismanDM. Metastatic extramammary Paget’s disease of scrotum responds completely to single agent trastuzumab in a hemodialysis patient: case report, molecular profiling and brief review of the literature. Case reports in oncological medicine. 2015;2015.10.1155/2015/895151PMC432283025692060

[19] BarrettT, WilhiteSE, LedouxP, EvangelistaC, KimIF, TomashevskyM, et al. NCBI GEO: archive for functional genomics data sets—update. 2012;41(D1):D991–D5.10.1093/nar/gks1193PMC353108423193258

[20] SongY, Guerrero-JuarezCF, ChenZ, TangY, MaX, LvC, et al. The Msi1-mTOR pathway drives the pathogenesis of mammary and extramammary Paget’s disease. Cell Res. 2020;30(10):854–72. doi: 10.1038/s41422-020-0334-5 32457396PMC7608215

[21] BarrettT, WilhiteSE, LedouxP, EvangelistaC, KimIF, TomashevskyM, et al. NCBI GEO: archive for functional genomics data sets—update. Nucleic Acids Res. 2012;41(D1):D991–D5.2319325810.1093/nar/gks1193PMC3531084

[22] ShermanBT, TanQ, CollinsJR, AlvordWG, RoayaeiJ, StephensR, et al. The DAVID Gene Functional Classification Tool: a novel biological module-centric algorithm to functionally analyze large gene lists. Genome Biol. 2007;8(9):1–16. doi: 10.1186/gb-2007-8-9-r183 17784955PMC2375021

[23] CvMering, Huynen M, Jaeggi D, Schmidt S, Bork P, Snel B. STRING: a database of predicted functional associations between proteins. Nucleic Acids Res. 2003;31(1):258–61. doi: 10.1093/nar/gkg034 12519996PMC165481

[24] ClineMS, SmootM, CeramiE, KuchinskyA, LandysN, WorkmanC, et al. Integration of biological networks and gene expression data using Cytoscape. Nat Protoc. 2007;2(10):2366. doi: 10.1038/nprot.2007.324 17947979PMC3685583

[25] TangZ, LiC, KangB, GaoG, LiC, ZhangZ. GEPIA: a web server for cancer and normal gene expression profiling and interactive analyses. Nucleic Acids Res. 2017;45(W1):W98–W102. doi: 10.1093/nar/gkx247 28407145PMC5570223

[26] GriffithM, GriffithOL, CoffmanAC, WeibleJV, McMichaelJF, SpiesNC, et al. DGIdb: mining the druggable genome. Nat Methods. 2013;10(12):1209–10. doi: 10.1038/nmeth.2689 24122041PMC3851581

[27] KuhnM, von MeringC, CampillosM, JensenLJ, BorkP. STITCH: interaction networks of chemicals and proteins. Nucleic Acids Res. 2007;36(suppl_1):D684–D8. doi: 10.1093/nar/gkm795 18084021PMC2238848

[28] ScarbroughCA, VrableA, CarrDR. Definition, Association with Malignancy, Biologic Behavior, and Treatment of Ectopic Extramammary Paget’s Disease: A Review of the Literature. The Journal of clinical and aesthetic dermatology. 2019;12(8):40. 31531170PMC6715119

[29] NgL, YipS, TanP. Extramammary Paget’s disease of scrotum. Urology. 2001;58(1):105. doi: 10.1016/s0090-4295(01)00976-1 11445493

[30] WangZ, LuM, DongGQ, JiangYQ, LinMS, CaiZK, et al. Penile and Scrotal Paget’s disease: 130 Chinese patients with long‐term follow‐up. BJU Int. 2008;102(4):485–8. doi: 10.1111/j.1464-410X.2008.07575.x 18336601

[31] ZampognaJC, FlowersFP, RothWI, HasseneinAM. Treatment of primary limited cutaneous extramammary Paget’s disease with topical imiquimod monotherapy: two case reports. J Am Acad Dermatol. 2002;47(4):S229–S35. doi: 10.1067/mjd.2002.126584 12271284

[32] WengS, ZhuN, LiD, ChenY, TanY, ChenJ, et al. Clinical Characteristics, Treatment, and Prognostic Factors of Patients With Primary Extramammary Paget’s Disease (EMPD): A Retrospective Analysis of 44 Patients From a Single Center and an Analysis of Data From the Surveillance, Epidemiology, and End Results (SEER) Database. Frontiers in oncology. 2020;10:1114. doi: 10.3389/fonc.2020.01114 32983958PMC7477308

[33] ChungPH, KamppJT, VoelzkeBB. Patients’ experiences with extramammary Paget disease: an online pilot study querying a patient support group. Urology. 2018;111:214–9. doi: 10.1016/j.urology.2017.08.045 28893632

[34] YangWJ, KimDS, ImYJ, ChoKS, RhaKH, ChoNH, et al. Extramammary Paget’s disease of penis and scrotum. Urology. 2005;65(5):972–5. doi: 10.1016/j.urology.2004.12.010 15882734

[35] HwangB-J, AdhikaryG, EckertRL, LuA-L. Chk1 inhibition as a novel therapeutic strategy in melanoma. Oncotarget. 2018;9(54):30450. doi: 10.18632/oncotarget.25765 30100999PMC6084399

[36] DinarinaA, PerezLH, DavilaA, SchwabM, HuntT, NebredaAR. Characterization of a new family of cyclin-dependent kinase activators. Biochem J. 2005;386(2):349–55. doi: 10.1042/BJ20041779 15574121PMC1134800

[37] GuhaM. Cyclin-dependent kinase inhibitors move into Phase III. Nature reviews Drug discovery. 2012;11(12):892. doi: 10.1038/nrd3908 23197022

[38] IzadiS, NikkhooA, Hojjat-FarsangiM, NamdarA, AziziG, MohammadiH, et al. CDK1 in breast cancer: implications for theranostic potential. Anti-Cancer Agents in Medicinal Chemistry (Formerly Current Medicinal Chemistry-Anti-Cancer Agents). 2020;20(7):758–67. doi: 10.2174/1871520620666200203125712 32013835

[39] BednarekK, KiwerskaK, SzaumkesselM, BodnarM, Kostrzewska-PoczekajM, MarszalekA, et al. Recurrent CDK1 overexpression in laryngeal squamous cell carcinoma. Tumor Biol. 2016;37(8):11115–26. doi: 10.1007/s13277-016-4991-4 26912061PMC4999469

[40] WuCX, WangXQ, ChokSH, ManK, TsangSHY, ChanACY, et al. Blocking CDK1/PDK1/β-Catenin signaling by CDK1 inhibitor RO3306 increased the efficacy of sorafenib treatment by targeting cancer stem cells in a preclinical model of hepatocellular carcinoma. Theranostics. 2018;8(14):3737. doi: 10.7150/thno.25487 30083256PMC6071527

[41] LiuY, DeguchiY, TianR, WeiD, WuL, ChenW, et al. Pleiotropic effects of PPARD accelerate colorectal tumorigenesis, progression, and invasion. Cancer Res. 2019;79(5):954–69. doi: 10.1158/0008-5472.CAN-18-1790 30679176PMC6397663

[42] MalumbresM, BarbacidM. Cell cycle, CDKs and cancer: a changing paradigm. Nature reviews cancer. 2009;9(3):153–66. doi: 10.1038/nrc2602 19238148

[43] CarbottaG, SallustioP, PresteraA, LaforgiaR, LobascioP, PalascianoN. Perineal Paget’s disease: A rare disorder and review of literature. Annals of medicine and surgery. 2016;9:50–2. doi: 10.1016/j.amsu.2016.06.012 27408714PMC4930340

[44] LiuG, LiC, ZhenH, ZhangZ, ShaY. Identification of prognostic gene biomarkers for metastatic skin cancer using data mining. Biomedical Reports. 2020;13(1):22–30. doi: 10.3892/br.2020.1307 32494360PMC7257933

[45] OttoT, SicinskiP. Cell cycle proteins as promising targets in cancer therapy. Nature Reviews Cancer. 2017;17(2):93. doi: 10.1038/nrc.2016.138 28127048PMC5345933

[46] GorlovI, OrlowI, RingelbergC, HernandoE, ErnstoffMS, ChengC, et al. Identification of gene expression levels in primary melanoma associated with clinically meaningful characteristics. Melanoma Res. 2018;28(5):380. doi: 10.1097/CMR.0000000000000473 29975213PMC6448582

